The article "Insulators' Identification and Missing Defect Detection in Aerial Images Based on Cascaded YOLO Models" was published in 2022. Journal: Comput Intell Neurosci.

# Insulators' Identification and Missing Defect Detection in Aerial Images Based on Cascaded YOLO Models

**DOI:** 10.1155/2022/7113765

**Published:** 2022-08-17

**Authors:** Jingjing Liu, Chuanyang Liu, Yiquan Wu, Zuo Sun, Huajie Xu

**Affiliations:** ^1^College of Mechanical and Electrical Engineering, Chizhou University, Chizhou 247000, China; ^2^College of Electronic and Information Engineering, Nanjing University of Aeronautics and Astronautics, Nanjing 211106, China

## Abstract

Insulators identification and their missing defect detection are of paramount importance for the intelligent inspection of high-voltage transmission lines. As the backgrounds are complex, some insulators may be occluded, and the missing defect of the insulator is so small that it is not easily detected from aerial images with different backgrounds. To address the above issues, in this study, a cascaded You Only Look Once (YOLO) models are mainly explored to perform insulators and their defect detection in aerial images. Firstly, the datasets used for insulators location and missing defect detection are created. Secondly, a new model is proposed to locate the position of insulators, which is improved in the feature extraction network and multisacle prediction network based on previous YOLOv3-dense model. An improved YOLOv4-tiny model is used to conduct missing defect detection on the detected insulators. And then, the proposed YOLO models are trained and tested on the built datasets, respectively. Finally, the final models are cascaded for insulators identification and their missing defect detection. The average precision of missing defect detection can reach 98.4%, which is 5.2% higher than that of faster RCNN and 10.2% higher than that of SSD. The running time of the cascaded YOLO models for missing defect detection can reach 106 frames per second. Extensive experiments demonstrate that the proposed deep learning models achieve good performance in insulator identification and its missing defect detection from the inspection of high-voltage transmission lines.

## 1. Introduction

With the continuous and rapid development of electric power in China, the total mileage of transmission lines also increases rapidly. The inspection of high-voltage transmission lines by an unmanned aerial vehicle (UAV) has attracted growing attentions in the power grid [1–3]. Conducting the regular inspection of key electrical equipment in high-voltage transmission lines is an effective way to ensure the safe and stable operation of the power grid [4], as shown in Figure 1(a). The aerial images captured by UAV consist of many different electrical equipment, e.g., insulator, antivibration hammers, and clamp are encircled by rectangular boxes with different colors. Specially, an insulator is an extremely important electrical equipment in high-voltage transmission lines, which plays the dual roles of mechanical support and electrical insulation [5, 6]. However, with the insulator's perennial exposure to wind, sun, and rain, coupled with snow and ice coverage and other adverse weather effects, the missing defect of insulator in transmission lines is inevitable, as shown in Figure 1(b). The missing defect of the insulator is encircled by a blue ellipse. Statistically, most of the power grid accidents are caused by the missing defect of the insulator, and therefore, it is of great significance to automatically and timely perform insulators' identification and their missing defect detection in high-voltage transmission lines [7, 8].

The article "Insulators' Identification and Missing Defect Detection in Aerial Images Based on Cascaded YOLO Models" was published in 2022. Journal: Comput Intell Neurosci.

Some scholars have committed to research on insulators and their missing defect detection in transmission lines, and many valuable research results have been obtained though target detection algorithms [9–14]. Commonly, according to whether it is necessary to manually design features, target detection algorithms can be divided into the traditional image processing method and the method based on deep learning [15]. The traditional method is composed of three parts, which are as follows: regions of interest (RoI) selection of different scales and widths, feature extraction, and target classification. Among them, the selection of RoI mostly uses the sliding window-based method. The manual designing method is the generally used manner for feature extraction (e.g., color feature, texture feature, scale invariant feature transform (SIFT), histogram of gradient (HOG), etc.). The support vector machine (SVM) and AdaBoost are the mainly used classifiers. Nevertheless, there are some disadvantages in the traditional method, such as the time-consuming nature and redundancy of the sliding window-based method, the manually designed feature is not robust to different environments, the computing ability is limited, and the processing ability of big data information is poor. Additionally, insulator aerial images are usually captured under complex backgrounds. Because of different shooting distances and angles, insulators and their missing defect are diverse, and they appear in different shapes. Consequently, in the practical applications, it is difficult for the traditional target detection method to recognize insulators and their missing defect in high-voltage transmission lines.

In the past decade, deep learning has made significant progress and become popular in the field of target detection, image classification, semantic segmentation, and so on [16–18]. Compared with the traditional target detection method, the method based on deep learning utilizes a nonlinear model to transform the low-level feature into high-level feature layer by layer and can automatically learn the useful features of the target, which have powerful learning and characterization capabilities, showing a strong advantage in feature extraction. Deep learning achieves the state-of-the-art performance in target detection by means of deep convolutional neural networks (DCNNs), which can represent the input image into high-dimensional feature space [19]. The development of deep learning has greatly promoted target detection, and target detection based on deep learning has become one of the research hotspots in the field of computer vision today. To improve the generalization performance of DCNNs, many excellent network structures of deep learning are proposed, particularly, LeNet, AlexNet, VGGNet, GoogleNet, ResNet, Densely Connected Convolutional Networks (DenseNet), and so on.

The article "Insulators' Identification and Missing Defect Detection in Aerial Images Based on Cascaded YOLO Models" was published in 2022. Journal: Comput Intell Neurosci.

Currently, deep learning algorithms used for target detection are generally divided into two categories, one-stage algorithm based on regression, and two-stage algorithm based on region proposal. Specifically, the two-stage algorithm divides the target detection problem into two steps. First of all, the candidate regions are selected from the input image, and then the classification and regression are performed on the selected candidate regions. The representative algorithms of two-stage are faster regions with convolutional neural networks (faster R-CNN) [20–24], region-based fully convolutional networks (R-FCN) [25], mask R-CNN [26], and cascade R-CNN [27–29]. The application research of electrical equipment detection in transmission lines based on two-stage target detection algorithms is shown in Table 1. The two-stage algorithm performs well on large-scale datasets, however, such an algorithm needs a large number of calculations and runs slowly. Hence, it is difficult to achieve the effect of real-time detection.

To improve real-time detection performance while ensuring accuracy, one-stage algorithms represented by YOLO [30–32] and single shot multibox detector (SSD) [33] have emerged. One-stage algorithms are regression-based target detection networks, which use DCNNs to extract features and directly realize classification and regression to obtain the category probability and location information of the target. The two-stage algorithms are the representatives of accuracy, which can fully learn the features of the target because they obtain the candidate regions in advance, however, the structures of networks are complex, and the detection speed is slow. Hence, they are not suitable for real-time applications, while one-stage algorithms are the representatives of speed, which can meet the requirements of application scenarios for real-time detection. Consequently, one-stage algorithms have a high application research value for insulator identification, and many satisfactory detection results are obtained by the use of one-stage algorithms [34–42]. In the work of [38], a novel SSD algorithm is proposed to recognize and localize insulators in visible light images. To realize multisize insulator detection in the background interference with high precision and low time cost, auxiliary convolutional feature layers are employed to VGG-16 network to replace the fully connected layers. Experimental results show that the mean running time of per image is 0.03 s, which is much faster than that of faster R-CNN (0.11 s per image). In the work of Tian [39], a deep learning architecture is proposed to automatically detect insulator faults in aerial images. Firstly, the SSD algorithm is utilized to detect the position of insulators. Then, DenseNet is used to determine the category of the detected insulators. Finally, experiments are conducted on the testing dataset. The precision of insulator detection and classification have reached 0.95 and 0.98, respectively. Compared with the YOLO algorithms, the detection speed of the SSD algorithm needs to be farther improved. To achieve multiple sizes of insulator detection in aerial images with complicated backgrounds, in the work of [40], three dense blocks are added to YOLOv3 to enhance feature propagation and reuse. The average precision of the modified YOLOv3 (YOLOv3-dense) model is 94.47%, and the average running time of per image can reach 8.5 ms, however, the modified model can only perform the localization detection of insulators, which is not used for the research of insulator defect detection. In [41], a deep neural network model is proposed to improve the accuracy and robustness of insulator detection in high-voltage transmission lines. The YOLOv3 model based on the backbone network of ResNet 50 is used to locate the position of insulator, and then the Grab-cut algorithm and the adaptive morphology method are used to perform insulator defect detection. Although the average running time of the YOLOv3 model can reach 0.02 s per image, it is difficult for the traditional image processing method to realize insulator defect detection in aerial images with diverse background interference. In [42], a cross stage partial dense YOLO (CSPD-YOLO) model is proposed for insulator defect detection, which achieves a good effect on the detection of the missing defect. Since the number of insulator defects is much lesser than that of the insulator, if the model is used for both insulators and their defect detection, it will lead to class imbalance [43].

The article "Insulators' Identification and Missing Defect Detection in Aerial Images Based on Cascaded YOLO Models" was published in 2022. Journal: Comput Intell Neurosci.

In summary, as the two-stage algorithms are hard to train and difficult to deploy on the embedded devices, it can thus be concluded that one-stage algorithms have the potential to meet the requirements of real-time detection, and the application of YOLO models on high-voltage transmission lines automatic inspection have very considerable prospects. To perform both insulator identification and missing defect detection in aerial images from high-voltage transmission lines, based on the previous work [40], and inspired by the deep learning architectures [27–29], this paper proposed a cascaded YOLO models (improved YOLOv3-dence and YOLOv4-tiny) for insulators' identification and their missing defect detection in aerial images. Specifically, improved YOLOv3-dense model is used to locate the insulators, and then the detected region of insulators is set as RoI area. Next, the improved YOLOv4-tiny model is employed to perform missing defect detection on RoI area.

The rest of this paper is organized as follows: Section 1 reports the related works of insulator identification and defect detection in aerial images.  Section 2 describes the proposed method in details.  Section 3 exhibits and discusses the experimental results and analysis of the proposed method. Finally, the conclusion and future work are shown in Section 4.

## 2. Materials and Methods

Since Hinton proposed the use of neural networks to automatically learn high-level feature in multimedia data, target detection based on deep learning has developed rapidly in the field of computer vision. Deep learning aims to locate the target of interest from the image, accurately determine the category of each target, and give the bounding box of each target. To obtain richer feature representation of target, on the one hand, large-scale image databases, such as ImageNet and COCO, are created. On the other hand, the commonly used backbone networks (e.g., VGGNet, GoogleNet, ResNet, etc.) are exploited to deepen DCNNs, promoting the accuracy and execution efficiency of target detection greatly. Recently, methods based on deep learning are widely used in the fields of video surveillance, intelligent transportation, the automatic driving of vehicles, pedestrian detection, face identification, robot navigation, and so on. Inspired by these state-of-the-art works, it is worth studying how to use deep learning algorithms for insulators' identification and their missing defect detection in UAV aerial images.

Cascaded deep learning models are designed to automatically detect insulators and their missing defects in complex aerial images. The improved YOLOv3-dense model and YOLOv4-tiny model are cascaded, which transforms insulator identification and missing defect detection to a two-level detection problem, directly uses improved YOLOv3-dense model to locate the position of insulator, and then improved YOLOv4-tiny model is used to perform the defect detection on the insulator. The entire architecture of the proposed method is shown in Figure 2. Firstly, insulator aerial images captured by UAV are used to construct the “CCIN_detection” (Chinese Composite INsulator) dataset [40], which is divided into the training dataset, testing dataset, and “InSF-detection” (Insulator Fault, InSF) dataset [42]. Secondly, the training dataset is utilized to train the improved YOLOv3-dense model for locating the insulator position, and the “InSF-detection” dataset is used to train the improved YOLOv4-tiny model for missing defect detection. The final models for insulator recognition and missing defect detecting are obtained after training. Finally, to verify the effectiveness of the proposed method, the final detection models are cascaded to perform insulator identification and missing defect detection on the testing dataset.

The article "Insulators' Identification and Missing Defect Detection in Aerial Images Based on Cascaded YOLO Models" was published in 2022. Journal: Comput Intell Neurosci.

### 2.1. Insulators' Identification

Insulator aerial images captured by UAV usually include complex backgrounds, such as river, farmland, power tower, building, and so on. In addition, since the characteristics are of multiangle and multiscale, the sizes of insulator are extremely diverse, resulting in difficult-to-recognize insulators in aerial images. Therefore, how to effectively extract and locate insulators in aerial images with complex background is very important. In our previous work [40], the YOLOv3-dense model (three dense blocks are adopted to the feature extraction network of the YOLOv3 model) is proposed to recognize the multisize of insulators amid diverse background interference. Experimental results conducted on the testing set of CCIN_detection show that the average precision (AP) value of the YOLOv3-dense model can reach 94.47%, which is higher than that of the YOLOv2 model (83.43%) and YOLOv3 model (90.31%). Although the experimental results verify that our proposed YOLOv3-dense model can effectively recognize insulators from the complex backgrounds, we decided to explore a new DCNN model, which is more accurate than the previous YOLOv3-dense model. To improve the accuracy of insulator identification, this section mainly focuses on the improvement of the feature extraction network and feature fusion based on YOLOv3-dense model. The entire structure of the proposed model is shown in Figure 3, which is made of feature extraction network, multiscale prediction network, and detection network.

The article "Insulators' Identification and Missing Defect Detection in Aerial Images Based on Cascaded YOLO Models" was published in 2022. Journal: Comput Intell Neurosci.

#### 2.1.1. Feature Extraction Network of the Proposed Model

The depth of DCNNs is very important to the detection performance of the deep learning model. The deeper network can extract high-efficiency features for targets identification, however, the detection accuracy of the model will quickly reach saturation as the network depth increases, and it even begins to decline rapidly. To solve the problem of network degradation, residual network (ResNet) is proposed by He et al. [44], so that the network with hundreds of layers can be trained. The main expression of ResNet is defined in formula (1).

(1) $$\begin{array}{c} x_{l}=H_{l}\left(x_{l-1}\right)+x_{l-1}, \end{array}$$

where *l* denotes the layer of DCNNs, *x*_*l*_ indicates the output of layer *l*, and *H*_*l*_ represents the nonlinear transformation of *x*_*l*−1_. In the ResNet module, the Conv (1 × 1) and Conv (3 × 3) are mainly employed. Conv (1 × 1) is used for compression feature representation, and Conv (3 × 3) is utilized for feature extraction.

To effectively reduce the parameters of the network model while keeping the low-level feature in the high-level layers as much as possible, the architecture of DenseNet is proposed by Huang et al. [45], which uses the dense connection between the layers to achieve information integration, avoiding the loss of feature information and the disappearance of gradients, so that the network can learn more features between different levels and improve the detection accuracy to a certain extent. The feed-forward manner is adopted to DenseNet to connect each layer to every other layer. In other words, the layer *l* receives all the features of the previous *l* − 1 layers as an input. The formula is defined as follows:

(2) $$\begin{array}{c} x_{l}=H_{l}\left(\left[x_{0},x_{1},\ldots ,x_{l-1}\right]\right), \end{array}$$

where [*x*_0_, *x*_1_,…, *x*_*l*−1_] denotes the output feature maps of layers *x*_0_, *x*_1_,…, *x*_*l*−1_ spliced in series. Moreover, the transform function *H*_*l*_ is a nonlinear function BN-ReLU-Conv (1 × 1)-BN-ReLU-Conv (3 × 3), which is a combination of batch normalisation (BN), rectified linear unit (ReLU), and convolutional (Conv).

To further improve the feature extraction network of YOLOv3-dense, CSPNet is adopted to the YOLOv3-dense model in this paper. CSPNet is a new type of backbone network proposed by Wang et al. [46] in 2020, which can be used to enhance the learning ability of DCNNs, maintain accuracy while being lightweight, reduce the computational bottlenecks, and reduce the cost of memory. In the structure of CSPNet, the feature maps of input layer are split into two parts: the first part is actually to yield a large residual edge, which is directly connected to the end after one convolutional operation. The latter is the main feature extraction part, which goes through a residual block, i.e., the number of channels is adjusted by Conv (1 × 1). Then, feature extraction is enhanced by Conv (3 × 3). The output is concatenated with the small residual edge, and finally, the number of channels is adjusted to be the same as the first part after the Conv (1 × 1) operation. The feature extraction network of the proposed model is shown in Table 2.

The article "Insulators' Identification and Missing Defect Detection in Aerial Images Based on Cascaded YOLO Models" was published in 2022. Journal: Comput Intell Neurosci.

As shown in Table 2, the feature extraction network of the proposed model can be divided into six parts, as follows: a Conv (3 × 3) is used for feature (416 × 416) extraction in the first part. A cross-stage partial convolution and one residual module are used for feature (208 × 208) extraction in the second part. A cross-stage partial convolution and two residual modules are utilized for feature (104 × 104) extraction in the third part. From the forth part to the sixth part, a cross-stage partial convolution, four dense modules, and four residual modules are employed for effective feature (52 × 52, 26 × 26, 13 × 13) extraction, as shown in Figure 4. Specifically, the input feature maps are (104 × 104 × 128) in the fourth part—Conv (256 × 1 × 1), Conv (256 × 3 × 3/2), four dense modules, four residual modules, Conv (128 × 1 × 1), and Conv (256 × 1 × (1) are used to extract feature (52 × 52). Firstly, Conv (256 × 3 × 3/(2) is used to compress image dimensions, and the feature maps (52 × 52 × 256) are obtained. Secondly, one part of feature maps (52 × 52 × 256) through Conv (256 × 1 × 1) to yield a large residual edge, and the other part of feature maps (52 × 52 × 256) is the main feature extraction part, which goes through four dense modules and four residual modules for feature extraction. During the process of feature extraction, the number of channels is adjusted to 128 through Conv (128 × 1 × 1), and BN-ReLU-Conv (32 × 1 × 1)-BN-ReLU-Conv (32 × 3 × (3) are applied to each dense module for feature extraction. Then, the four residual modules are used to continue extracting feature. Finally, the feature maps (52 × 52) generated from the two parts are concatenated, and then the number of channels is adjusted to 256 through Conv (256 × 1 × (1) to obtain the output feature maps (52 × 52 × 256). Similarly, the input feature maps are (52 × 52 × 256) in the fifth part—Conv (512 × 1 × 1), Conv (512 × 3 × 3/2), four dense modules, four residual modules, Conv (256 × 1 × 1), and Conv (512 × 1 × (1) are used to extract feature (26 × 26). BN-ReLU-Conv (64 × 1 × 1)-BN-ReLU-Conv (64 × 3 × (3) are employed to each dense module for feature extraction. The feature maps (26 × 26) generated from the two parts are concatenated, and then the number of channels is adjusted to 512 through Conv (512 × 1 × (1) to obtain the output feature maps (26 × 26 × 512). In the sixth part—Conv (1024 × 1 × 1), Conv (1024 × 3 × 3/2), four dense modules, four residual modules, Conv (512 × 1 × 1), and Conv (1024 × 1 × (1) are used to extract feature (13 × 13). BN-ReLU-Conv (128 × 1 × 1)-BN-ReLU-Conv (128 × 3 × (3) are applied to each dense module for feature extraction. The feature maps (13 × 13) generated from the two parts are concatenated, and then the number of channels is adjusted to 1024 through Conv (1024 × 1 × (1) to yield the output feature maps (13 × 13 × 1024).

The article "Insulators' Identification and Missing Defect Detection in Aerial Images Based on Cascaded YOLO Models" was published in 2022. Journal: Comput Intell Neurosci.

#### 2.1.2. Multiscale Pooling Module

The pooling operation is indispensable for DCNNs, which can reduce the size of images, while preserving the main information of the image as much as possible, so that the network model can focus more on the main feature. Spatial pyramid pooling (SPP) is a method proposed by He et al. [47] to solve the problem of images with different sizes input to the DCNNs, generating a fixed-size feature representation without considering the size or proportion of the input image. Different from the purpose of work [47], a structure of SPPNet is employed in this paper, aiming to obtain multiscale local features information and fuse them with global feature information to enrich the expressive ability of the feature maps, thereby improving the accuracy of target prediction.

To further obtain more local features, a multiscale pooling module is used in the last feature layer of the feature extraction network, as shown in Figure 5. Three max-pooling layers of different kernel sizes (5 × 5, 9 × 9, 13 × 13) are used to obtain multiscale local feature maps, and then the local feature maps are concatenated with the input global feature maps. By the use of the multiscale pooling module, the receptive field of the last feature layer can be expanded. In addition, the richer local features information can be obtained, and the sensitivity of the target with different scales can be improved.

#### 2.1.3. Multiscale Prediction Network

In the previous YOLOv3-dense model, the effective feature maps (52 × 52, 26 × 26, 13 × 13) that corresponded to different levels of feature information are selected for feature fusion. As the span between these feature maps is very large, after multiple convolution operations, the feature at each level retains less feature information from other levels. As the number of network layers continues to deepen, the feature extraction of semantic information becomes better, however, with the enhancement of semantic information, the loss of detailed information (e.g., shape feature, color feature, texture feature, etc.) brings many negative effects on insulator localization, resulting in it being impossible to accurately locate the position of insulators. To enhance the feature representation and further realize feature reuse, the top-down and bottom-up fusion strategy [48] is employed to the multiscale prediction network. The structure of multiscale prediction network is shown in Figure 6.

The article "Insulators' Identification and Missing Defect Detection in Aerial Images Based on Cascaded YOLO Models" was published in 2022. Journal: Comput Intell Neurosci.

As shown in Figure 6, the process of multiscale prediction is as follows: firstly, the original image is subjected to feature extraction through the forward propagation of DCNNs. The size of the feature layers is gradually reduced, and the effective feature maps (C3, C4, and C5) are extracted. Secondly, convolutional operation and SPP are performed on feature maps C5 to generate feature maps P3, and then the feature maps P3 are fused with feature maps C4 via convolutional operation and up-sampling to obtain feature maps P2, while the feature maps P2 are fused with feature maps C3 via convolutional operation and up-sampling to yield feature maps P1. Finally, the convolutional operation is performed on feature maps P1 to generate feature maps N1, and then the feature maps N1 are fused with the feature maps P2 via convolutional operation and down-sampling to obtain feature maps N2, while the feature maps N2 are fused with the feature maps P3 via convolutional operation and down-sampling to generate feature maps N3. The feature maps N1, N2, and N3 are connected to the residual modules for feature (52 × 52, 26 × 26, 13 × 13) prediction, respectively. The feature maps from P3 to P1 is a top-down process. The high-level feature that contains more semantic information is fused with low-level feature through up-sampling, and the feature maps from N1 to N3 is a bottom-up process. The detailed information of low-level feature and the semantic information of high-level feature are retained for more accurate locating prediction.

### 2.2. Missing Defect Detection

In the process of transmission lines inspection based on UAV, it is commonly faced with complex scenes and changeable climate, which makes it difficult to inspect high-voltage transmission lines. Furthermore, there are still safety distance restrictions for UAV to fly along high-voltage transmission lines, resulting in the electrical equipment being captured by UAV accounts for a very small proportion to the whole image. Since most of insulator missing defect area is relatively small, the information of the defect area will be lost after multiple convolutional operation. As a result, the one-stage algorithm will not be able to effectively detect the position of insulator missing defect. In this work, cascaded deep learning models are employed for insulator identification and missing defect detection. Firstly, the first detection model (improved YOLOv3-dense model) detailed in section 2.1 is adopted to locate the position of insulators in aerial images. Then, the localization of insulator detected by the proposed model is set as the RoI area. Finally, the second detection model (improved YOLOv4-tiny) is used to perform missing defect detection on the RoI area.

The article "Insulators' Identification and Missing Defect Detection in Aerial Images Based on Cascaded YOLO Models" was published in 2022. Journal: Comput Intell Neurosci.

YOLOv4-tiny network is an abbreviated version of YOLOv4 model, which uses a more lightweight backbone network to extract image features, simplifies the feature fusion part of the neck, reduces the output branch of the head, and improves the detection speed of the network. More importantly, the memory usage of the final weights for the YOLOv4-tiny model is less than 30 MB, so that it is suitable for running on mobile or embedded devices for real-time detection. To improve the detection accuracy of insulator missing defect, we improve YOLOv4-tiny on the multiscale prediction network. The feature (52 × 52) detection head (in the red rectangular box) is added to the prediction network, and the entire structure of improved. The YOLOv4-tiny model is shown in Figure 7.

## 3. Experiments' Results and Discussion

### 3.1. Experimental Environment

In this study, we conduct training and testing by the use of the deep learning framework Dark-net [49]. A server equipped with hardware and software is constructed to evaluate the proposed method. The basic configuration of the hardware platform is as follows: an Intel (R) Core (TM) i9-9900K CPU and an NVIDIA GeForce GTX 3080 GPU. The basic configuration of the software platform is as follows: Windows 10 as the basic operating system, Opencv3.4.0 and Visual Studio 2017 as the graphics processing tools, CUDA 11.1 as parallel computing architecture, and cuDNN 8.0.5 as DCNNs acceleration library. The detail information of experimental environment is shown in Table 3.

### 3.2. Dataset Preparation

There is no known existing image dataset toward the missing defect estimation of the insulator. Hence, data collection is a significant part of the effort for this paper. For a fair comparison with YOLOv3-dense model, the proposed model described in section 2.1 is trained on the CCIN_detection dataset. First of all, we collect 5000 aerial images in total, which are more diverse and contain more common aerial scenes compared with the images in CPLID (Chinese Power Line Insulator Dataset) [27]. Next, all the images are resized to the same size of 416 × 416 pixels, and the LabelImg tool is utilized to label the ground-truth for all the insulator images. Finally, we randomly select 3000 images as a training set, and the other 2000 images are assigned to be a testing set.

The article "Insulators' Identification and Missing Defect Detection in Aerial Images Based on Cascaded YOLO Models" was published in 2022. Journal: Comput Intell Neurosci.

Since the number of insulator missing defect is usually less than that of insulators in aerial images and the position of the missing defect is uncertain, it is impossible to get enough missing defect samples of real scenes for conducting insulator missing defect detection. To address the above issues, the image processing tool of Photoshop is used to obtain simulated missing defect samples. Ultimately, the InSF-detection dataset with 1331 aerial images is created, in which 809 images are set to be a training set, while the other 522 images are set to be a testing set. The relevant information of two datasets is shown in Table 4.

### 3.3. Quantitative and Qualitative Analysis

To evaluate the effectiveness of the proposed model described in Section 2.1, extensive experiments are conducted on the proposed model and the compared models (YOLOv3 and YOLOv3-dense). For a fair comparison, the proposed model, YOLOv3, and YOLOv3-dense are trained and tested on the same dataset CCIN_detection. During the process of training, the number of iterations is set to be 38,000, the initial value of the learning rate is set as 0.001, decay = 0.005, momentum = 0.9, saturation = 1.5, hue = 0.1, exposure = 1.5, batch size = 64, and subdivision = 16, respectively.

In addition, average precision (AP), precision (P), and recall (R) are used to verify the effects of the proposed model quantitatively. The true positive (TP), false positive (FP), true negative (TN), and false negative (FN) are four common types used to evaluate the binary classification model. The definitions of TP, FP, TN, and FN are shown in Table 5. Among them, TP represents the number of samples where the detected category is consistent with the real target category, FP indicates the number of samples in which the detected target category is inconsistent with the real target category, TN represents the number of negative samples that is correctly classified, and FN indicates the number of samples in which the real target exists but has not been detected.

Precision (P) can be defined as the proportion of all correctly predicted targets to all the predicted targets, as shown in formula (3).

(3) $$\begin{array}{c} Precision\left(P\right)=\frac{\text{TP}}{\text{TP}+\text{FP}}. \end{array}$$

Recall (R) can be defined as the proportion of all correctly predicted targets to all the targets that should be predicted, as shown in formula (4).

(4) $$\begin{array}{c} Recall\left(R\right)=\frac{\text{TP}}{\text{TP}+\text{FN}}. \end{array}$$

The precision-recall (P-R) curve is usually used to evaluate the performance of deep learning model, which can be obtained by taking the recall value as the horizontal axe and precision value as the vertical axe. The AP value can be calculated by the area under the P-R curve, as shown in formula (5).

(5) $$\begin{array}{c} AP=\int_{0}^{1}P\left(R\right)\text{ d}R. \end{array}$$

The article "Insulators' Identification and Missing Defect Detection in Aerial Images Based on Cascaded YOLO Models" was published in 2022. Journal: Comput Intell Neurosci.

#### 3.3.1. Insulators' Identification Based on the Proposed YOLO Model

To evaluate the effect of insulators' identification, the proposed model and the compared models (YOLOv3 and YOLOv3-dense) are trained and then tested. The experimental effects (AP, precision, and recall) of three models for insulators' identification are listed in Table 6. Specifically, the AP values of three insulator identification models are as follows: YOLOv3 (90.3%), YOLOv3-dense (94.4%), and the proposed model (96.3%). It is found that the AP value of the proposed model is 6% higher than that of YOLOv3 and 1.9% higher than that of YOLOv3-dense, which demonstrates that the proposed detection model is more accurate than YOLOv3 and YOLOv3-dense. The precision values of the three insulator detection models are as follows: YOLOv3 (90%), YOLOv3-dense (94%), and the proposed model (96%). The precision value of the proposed detection model is 6% higher than that of YOLOv3 and 2% higher than that of YOLOv3-dense. The recall values of the three insulator detection models are as follows: YOLOv3 (91%), YOLOv3-dense (96%), and the proposed model (97%). The recall value of the proposed detection model is 6% higher than that of YOLOv3 and 1% higher than that of YOLOv3-dense. It can be concluded that the proposed model is more advantageous than YOLOv3 and YOLOv3-dense for insulators' identification.

To further analyze the impact of the improved method proposed in this paper on the YOLOv3 model, ablation experiments are conducted. The algorithm in this paper is cut into five groups for training, respectively. The first group is the original YOLOv3 model, the second group is the feature extraction network structure of YOLOv3 changed to CSPNet, the third group is the multiscale pooling module (SPPNet) added to the previous group, the fourth group is the addition of multiscale prediction network (PANet) on the basis of the previous group, and the fifth group is the residual module used on the basis of the previous group, i.e., the fifth group is the algorithm proposed in this paper. Experimental results of the five groups are shown in Table 7.

It can be obtained from Table 7 for the first group of the experiment. The AP value of the original YOLOv3 model on insulators' identification is 90.3%, and the FPS (frames per second) is 125. For the second group of the experiment, because of the introduction of CSPNet, the AP value of the insulators' identification increases by 3.5%, and at the same time, the increase of FPS is 5. The cross-stage partial network enhances the learning ability of the convolutional network, eliminates most of the computational bottleneck structure, and reduces the memory consumption, thus improving the accuracy of detection and inference speed. For the third group of experiment, since the improved spatial pyramid pooling structure is added on the basis of the second group, although 2 FPS is sacrificed compared to the second group, the AP value increases by 1%, which shows that the improved spatial pyramid pooling structure is meaningful for improving the accuracy of model detection. For the fourth group of the experiment, since the path aggregation network is added on the basis of the third group, the AP on insulators identification can improve to a certain extent. It is because a bottom-up fusion path is added to the three effective feature layers, which further improves the detection effect of the prediction network. For the fifth group of experiment, the residual module is introduced on the basis of the fourth group. Compared with the fourth group, the AP value increases by 0.8%, especially compared with the original YOLOv3 model, which has a significant improvement as a whole. Meanwhile, the proposed model also achieves better real-time effect, and the FPS increases by 10 compared with YOLOv3. In summary, the improvement strategies proposed in this paper for YOLOv3 model are meaningful for improving the effects of insulators' identification in complex scenes.

The article "Insulators' Identification and Missing Defect Detection in Aerial Images Based on Cascaded YOLO Models" was published in 2022. Journal: Comput Intell Neurosci.

Insulator images captured by UAV usually contain complex backgrounds, e.g., river, farmland, power tower, building, sky, and so on. Moreover, the sizes of insulators in aerial image change significantly because of the different filming angles and distances in real-world applications. Some typical images with different backgrounds are selected to verify the accuracy of the proposed model in insulators' identification, as shown in Figure 8, which exhibit the experimental scenes with the background of river, farmland, power tower, building, and sky, respectively. Specifically, figure 8(a) demonstrate experimental results with river background interference in the aerial images. The river background is not complex. Two insulators under strong light and one insulator under occlusion condition are correctly predicted in the figures.  Figure 8(b) shows experimental results with farmland background interference in the aerial images. All the insulators of different sizes are correctly predicted in the figures. Experimental results with power tower background interference in the aerial images are exhibited in figure 8(c). The uncertainty of perspective and occlusion can easily occur in the aerial image. Although the background of the power tower is complex, all the insulators are predicted in the figures, including two heavily occluded insulators. Experimental results with building background interference in the aerial images are demonstrated in figure 8(d), insulators with large differences in sizes, and insulators similar to the background in color are accurately predicted in the figures.  Figure 8(e) shows experimental results with sky background interference in the aerial images. The sky background is simple compared with figures 8(a)–8(d). All the insulators with different sizes and shapes are accurately predicted in the figures. Therefore, it can be concluded that the proposed model achieves good performance in insulators' identification.

#### 3.3.2. Insulator Missing Defect Detection Based on Improved YOLOv4-Tiny

To evaluate the effect of insulator missing defect detection, YOLOv3-tiny, YOLOv3, and improved YOLOv4-tiny are trained and tested on the dataset InSF-detection. The experimental effects (AP, precision, recall, memory usage, and running time) of the three models for insulator missing defect prediction are listed in Table 8. Specifically, the AP values of the three network models are as follows: YOLOv3-tiny (89.6%), YOLOv3 (93.3%), and the improved YOLOv4-tiny (92.9%). The precision values of the three network models are as follows: YOLOv3-tiny (92%), YOLOv3 (94%), and the improved YOLOv4-tiny (94%). The Recall values of the three network models are as follows: YOLOv3-tiny (89%), YOLOv3 (94%), and the improved YOLOv4-tiny (89%). It is found that the AP value of the improved YOLOv4-tiny is just a little lower than that of YOLOv3. The memory usages of the three network models are as follows: YOLOv3-tiny (33 MB), YOLOv3 (240 MB), and the improved YOLOv4-tiny (24 MB), and the running times of the three network models are as follows: YOLOv3-tiny (4.5 ms), YOLOv3 (10 ms), and the improved YOLOv4-tiny (4 ms). It can be observed that improved YOLOv4-tiny not only takes up less memory usage but also has faster detection speed. Consequently, considering the AP values, memory usages, and running times, it can be concluded that the improved YOLOv4-tiny model is suitable to deploy on embedded devices for insulator defect detection.

Experimental results with different scenes conducted by improved YOLOv4-tiny model are shown in Figure 9. Figures 9(a)–9(d) demonstrate the experimental scenes with the background of river, farmland, power tower, and sky, respectively. From the figures 9(a)–9(d), it is found that all the insulators with a single-defect or multiple-defect are accurately detected in aerial images with different background interference by the improved YOLOv4-tiny model.

The article "Insulators' Identification and Missing Defect Detection in Aerial Images Based on Cascaded YOLO Models" was published in 2022. Journal: Comput Intell Neurosci.

#### 3.3.3. The Cascaded YOLO Models for Insulators Detection

To verify the accuracy and robustness of the proposed method, improved YOLOv3-dense model and YOLOv4-tiny model are cascaded to perform insulators' identification and their missing defect detection. The cascaded YOLO models, faster RCNN, and SSD are tested on the testing dataset of “CCIN_detection,” and YOLOv4, models in Literature [42, 50], faster RCNN, SSD, our proposed models are used for insulator missing defect detection on the testing dataset of “InSF-detection.” The AP, precision, recall, and FPS values of the six models for the insulator missing defect prediction are listed in Table 9. Concretely, the AP values of the six models are as follows: YOLOv4 (96.38%), model in [50] (96.5%), model in [42] (98.18%), Faster RCNN (93.2%), SSD (88.1%), and the cascaded YOLO models (98.40%). The precision values of the six models are as follows: YOLOv4 (98%), model in [50] (98%), model in [42] (99%), Faster RCNN (94%), SSD (85%), and the cascaded YOLO models (99%). The recall values of the six models are as follows: YOLOv4 (95%), model in Literature [50] (95%), model in [42] (98%), Faster RCNN (92%), SSD (89%), and the cascaded YOLO models (98%). The FPS values of the six models are as follows: YOLOv4 (100), model in [50] (100), model in [42] (91), Faster RCNN (35), SSD (78), and the cascaded YOLO models (106), respectively. Since insulator defect detection can be regarded as small target detection and the AP value of our proposed model is 98.4%, which is 5.2% higher than that of faster RCNN and 10.2% higher than that of SSD, our proposed model has good ability for small object detection. Simultaneously, the FPS value of our proposed model can reach 106, which is the biggest in the six models. Accordingly, it can be found that the cascaded YOLO models can be more advantageous than the faster RCNN, SSD, YOLOv4, and models in Literature [42, 50] in insulator missing defect prediction.

Some typical images with different scenes are selected to exhibit the visualization performance of the cascaded YOLO models, as shown in Figure 10. The experimental scenes with backgrounds of river, farmland, and power tower were exhibited in figures 10(a)–10(c), the experimental scene with the insulator's color being similar to the background is shown in Figure 10(d), and the experimental scene with the occlusion of insulator strings is demonstrated in Figure 10(e). Although the backgrounds are complex, the insulator's color is similar to the background, and part of the insulator strings are occluded. All the insulators and their defects are accurately detected by the cascaded YOLO models. Consequently, it may be concluded that the proposed method (improved YOLOv3-dense and YOLOv4-tiny are cascaded) can obtain good performance in insulators' identification and their missing defect detection in aerial images with complex backgrounds.

The article "Insulators' Identification and Missing Defect Detection in Aerial Images Based on Cascaded YOLO Models" was published in 2022. Journal: Comput Intell Neurosci.

## 4. Conclusions

This study presented cascaded YOLO models for insulators' identification and their missing defect detection in aerial images from high-voltage transmission lines. First of all, “CCIN_detection” dataset, including 5000 insulator images and “InSF-detection” dataset consisting of 1331 insulator defect images were created. After that, to improve the accuracy of insulator detection from complex background interference, the feature extraction network and multisacle prediction network were improved in our previous YOLOv3-dense model. Moreover, the detected area of insulator was set as RoI area, and improved YOLOv4-tiny model with three detection heads was used to perform missing defect detection on the RoI area. Finally, the improved YOLOv3-dense and YOLOv4-tiny models were carefully trained, and the final models were cascaded to conduct insulator identification and defect detection on the testing set. Extensive experiments were performed on the cascaded YOLO models and the compared models. The experimental results showed that the AP values of YOLOv3-dense, YOLOv3, and the improved YOLOv3-dense were 94.4%, 90.3%, and 96.3%, respectively, proving the proposed model was superior to YOLOv3 and YOLOv3-dense models. The AP value of the improved YOLOv4-tiny (92.6%) model was slightly lower than that of the YOLOv3 (93.3%) model. More importantly, the memory usage of the improved YOLOv4-tiny (24 MB) model was much less than that of YOLOv3 (240 MB) and YOLOv3-tiny (33 MB) models. The AP and FPS values of cascaded YOLO models for insulator missing defect detection could reach 98.40% and 106, which are higher than those of the compared models. Therefore, it can be concluded that the cascaded models can obtain good performance in insulators' identification and their missing defect detection in aerial images and have the potential of real-time inspection for high-voltage transmission lines.

For a future study, the samples of insulators and their missing defect should be collected and added to datasets “CCIN_detection” and “InSF-detection.” In addition, the proposed models should be adjusted to adapt to more types of insulator defect detection.

The article "Insulators' Identification and Missing Defect Detection in Aerial Images Based on Cascaded YOLO Models" was published in 2022. Journal: Comput Intell Neurosci.

## Figures and Tables

**Figure 1:** Aerial images captured by UAV: (a) different electrical equipment of transmission lines in the image (e.g., insulator, antivibration hammers, clamp, etc.) and (b) missing defect of insulator. (a) Aerial image with different electrical equipment. (b) Aerial image with missing defect of insulator.

**Figure 2:** Cascaded architecture for insulator identification and missing defect detection.

**Figure 3:** The entire structure of the proposed model.

**Figure 4:** The effective feature extraction parts of the proposed model.

**Figure 5:** The structure of SPPNet.

**Figure 6:** The structure of multiscale prediction network.

**Figure 7:** The entire structure of improved YOLOv4-tiny network.

**Figure 8:** Experimental results with different scenes conducted by the proposed model (from the first row to the fifth row show experimental scenes with the background of river, farmland, power tower, building, and sky, respectively). (a) Experimental scene with the background of a river, (b) experimental scene with the background of farmland, (c) experimental scene with the background of a power tower, (d) experimental scene with the background of a building, and (e) experimental scene with the background of the sky.

**Figure 9:** Experimental results with different scenes conducted by improved YOLOv4-tiny. (a) River background, (b) farmland background, (c) power tower background, and (d) sky background.

**Figure 10:** Experimental results with different scenes conducted by the cascaded models. (a) Experimental scene with a river in the background. (b) Experimental scene with a farmland in the background. (c) Experimental scene with a power tower in the background. (d) Experimental scene with the insulator's color being similar to the background. (e) Experimental scene with the occlusion of insulator strings.

**Table 1:** The application research of two-stage algorithms on electrical equipment detection.

Algorithm	Target detection	Detection effect
Faster R-CNN [20]	Insulators and their faults	Achieves a precision of 94% and a recall of 88%
Faster R-CNN [21]	Insulator detection	The average precision value reaches 0.818 using VGG-16
Faster R-CNN [22]	8 defects in transmission lines	The defects can be effectively and accurately identified
Faster R-CNN [23]	Insulator self-explosion defect	The identification rate reaches 89.0%
Faster R-CNN [24]	Insulator	The average precision at a level of 0.8 for 60 frames
R-FCN [25]	Cracked insulator detection	The average accuracy rate of 90.5%
Mask R-CNN [26]	Insulator identification and self-shattering detection	The mean average precision can be up to 1 for single-target images and 0.948 for multitarget images
LIN + DDN [27]	Insulator defect detection	Defect detection precision and recall are 0.91 and 0.96
Faster R-CNN + FCN [28]	Identification of insulator explosion	The faulted insulators can be effectively detected in highly cluttered images
Faster R-CNN + Res-Unet [29]	Insulator defect identification	The precision and recall are 91.9% and 95.7%

The article "Insulators' Identification and Missing Defect Detection in Aerial Images Based on Cascaded YOLO Models" was published in 2022. Journal: Comput Intell Neurosci.

**Table 2:** The feature extraction network of the proposed model.

Cross-stage partial		Type	Filters	Size	Output
		Convolutional	32	3 × 3/1	416 × 416 × 32
		Convolutional	64	3 × 3/2	

Conv (64 × 1 × 1)	1×	Convolutional	32	1 × 1/1	
		Convolutional	64	3 × 3/1	
		Residual			
		Convolutional	64	1 × 1/1	208 × 208 × 64
		Convolutional	128	3 × 3/2	

Conv (128 × 1 × 1)	2×	Convolutional	64	1 × 1/1	
		Convolutional	128	3 × 3/1	
		Residual			
		Convolutional	128	1 × 1/1	104 × 104 × 128
		Convolutional	256	3 × 3/2	
		Convolutional	128	1 × 1/1	

Conv (256 × 1 × 1)	4×	Convolutional	32	1 × 1/1	
		Convolutional	32	3 × 3/1	
		DenseNet			
	4×	Convolutional	128	1 × 1/1	
		Convolutional	256	3 × 3/1	
		Residual			
		Convolutional	256	1 × 1/1	52 × 52 × 256
		Convolutional	512	3 × 3/2	

Conv (512 × 1 × 1)		Convolutional	256	1 × 1/1	
	4×	Convolutional	64	1 × 1/1	
		Convolutional	64	3 × 3/1	
		DenseNet			
	4×	Convolutional	128	1 × 1/1	
		Convolutional	256	3 × 3/1	
		Residual			
		Convolutional	512	1 × 1/1	26 × 26 × 512
		Convolutional	1024	3 × 3/2	

Conv (1024 × 1 × 1)		Convolutional	256	1 × 1/1	
	4×	Convolutional	128	1 × 1/1	
		Convolutional	128	3 × 3/1	
		DenseNet			
	4×	Convolutional	512	1 × 1/1	
		Convolutional	1024	3 × 3/1	
		Residual			
		Convolutional	1024	1 × 1/1	13 × 13 × 1024

**Table 3:** The detail information of experimental environment.

Parameters	Configuration
Framework	Dark-net
CPU	Intel(R) Core (TM) i9-9900K, CPU/3.6 GHz,
Memory	RAM/32 G
GPU	Nvidia GeForce GTX 3080 (10G)
Operating system	Windows 10
Graphics processing tool	Open CV 3.4.0, visual Studio 2017
Accelerated environment	CUDA 11.1, cuDNN 8.0.5

**Table 4:** The relevant information of two datasets.

Dataset	Number of images	Training set	Testing set	Image size
CCIN_detection	5000	3000	2000	416 × 416
InSF-detection	1331	809	522	416 × 416

**Table 5:** The definition of TP, FP, TN, and FN.

Ground truth	Prediction result	Definition
Positive (1)	Positive (1)	TP
Positive (1)	Negative (0)	FN
Negative (0)	Positive (1)	FP
Negative (0)	Negative (0)	TN

**Table 6:** The experimental effects of three insulator identification models.

Networks	AP (%)	Precision (%)	Recall (%)
YOLOv3	90.3	90	91
YOLOv3-dense	94.4	94	96
Proposed model	96.3	96	97

The article "Insulators' Identification and Missing Defect Detection in Aerial Images Based on Cascaded YOLO Models" was published in 2022. Journal: Comput Intell Neurosci.

**Table 7:** Comparison of ablation experimental results.

Methods	CSPNet	SPPNet	PANet	Residual module	AP (%)	FPS
YOLOv3 (1)					90.3	125
YOLOv3 (2)	√				93.8	130
YOLOv3 (3)	√	√			94.8	128
YOLOv3 (4)	√	√	√		95.5	132
YOLOv3 (5)	√	√	√	√	96.3	135

**Table 8:** The experimental effects of three insulator missing defect detection models.

Networks	AP (%)	Precision (%)	Recall (%)	Memory usage (MB)	Running time (ms)
YOLOv3-tiny	89.6	92	89	33	4.5
YOLOv3	93.3	94	94	240	10
Improved YOLOv4-tiny	92.9	94	89	24	4

**Table 9:** The experimental effects of different networks.

Networks	AP (%)	Precision (%)	Recall (%)	FPS
YOLOv4	96.38	98	95	100
Literature [50]	96.5	98	95	100
Literature [42]	98.18	99	98	91
Faster RCNN	93.2	94	92	35
SSD	88.1	85	89	78
Our proposed models	98.40	99	98	106

## Data Availability

No data were used to support this study.
